This article has been retracted.

# Interference of the long noncoding RNA CDKN2B‐AS1 upregulates miR‐181a‐5p/TGFβI axis to restrain the metastasis and promote apoptosis and senescence of cervical cancer cells

**DOI:** 10.1002/cam4.2040

**Published:** 2019-03-18

**Authors:** Lihong Zhu, Quanhua Zhang, Shaoping Li, Shan Jiang, Jingjing Cui, Ge Dang

**Affiliations:** ^1^ Department of Obstetrics and Gynecology The First Affiliated Hospital of Xinxiang Medical University Xinxiang China; ^2^ Department of Surgery The First Affiliated Hospital of Xinxiang Medical University Xinxiang China

**Keywords:** CDKN2B‐AS1, cervical cancer, epithelial‐mesenchymal transition, senescence

## Abstract

Long noncoding RNA (lncRNA) CDKN2B‐AS1 has been shown to play a crucial role in the development as well as in the prognosis of various human cancers, including cervical cancer. However, the underlying mechanisms need to be further explored between CDKN2B‐AS1 and cervical cancer. In the present study, RT‐PCR showed that the mRNA level of CDKN2B‐AS1 was significantly upregulated while the miR‐181a‐5p was downregulated in cervical cancer cell lines. In addition, the interference of CDKN2B‐AS1 by shRNA resulted in the suppression of cell proliferation, invasion, migration and promotion of apoptosis and senescence, and either CDKN2B‐AS1 overexpression or miR‐181a‐5p showed reversed results. Further studies demonstrated that CDKN2B‐AS1 could directly interact with miR‐181a‐5p, and that there was an inverse correlation between miR‐181a‐5p and CDKN2B‐AS1. In addition, we found that TGFβI was a target of miR‐181a‐5p and could be downregulated by CDKN2B‐AS1 knockdown. Moreover, the in vivo experiments further demonstrated the contribution of CDKN2B‐AS1 in cervical cancer including tumor growth, apoptosis inhibition and senescence inhibition, and CDKN2B‐AS1 knockdown could inhibit the aforementioned activities. In summary, our study demonstrated that the CDKN2B‐AS1/miR‐181a‐5p/TGFβI axis might play a vital role in cervical cancer development.

## 1 INTRODUCTION

Cervical cancer is the second most commonly diagnosed cancer and the third leading cause of cancer death among females in less developed countries.^1^ Human papillomaviruses (HPVs) are the common etiologic risk factor of cervical cancer.^2^ Widespread implementation of Pap smear screening programs in recent years has decreased the incidence and mortality of cervical cancer in many countries. Despite this, cervical cancer remains to be a major public health problem.^3^ Major research efforts have focused on the identification of tumor‐specific markers for predicting the biological behavior of cervical cancers. Several long noncoding RNAs(lncRNAs), including CCAT2,^4^ MALAT‐1,^5^ MEG3,^6^ ZNRD1‐AS1,^7^ and HOTAIR,^8^ have been shown to modulate cervical cancer. These lncRNAs may represent potential prognostic markers for predicting the aggressiveness of cervical cancer. It is practical to clarify the molecular mechanisms underlying cervical carcinogenesis and progression, which is required to identify reliable prognostic markers of cervical cancer.

LncRNA CDKN2B anti‐sense RNA (CDKN2B‐AS1, also named ANRIL, a 3.8‐kb long noncoding RNA), has been verified to be upregulated in tumor tissue and function as a tumor‐promoting lncRNA in numerous malignancies, such as hepatocellular carcinoma,^9^ non‐small cell lung cancer,^10^ cervical cancer,^10^ ovarian cancer, and 11 bladder cancer.^12^ It has been reported to regulate tumor cell proliferation, invasion, migration, apoptosis and senescence.^11^, ^12^, ^13^ Moreover, CDKN2B‐AS1 is significantly upregulated in most of the tumor cancer cells, including cervical cancer.^14^ A previous study reported that CDKN2B‐AS1 contributed to cervical cancer recurrence and might have diagnostic value in cervical cancer.^14^ In addition, CDKN2B‐AS1 was reported to enhance the proliferation, invasion, migration, and reduce apoptosis and senescence of cervical cancer cells.^13^, ^14^ Abundance of articles found that CDKN2B‐AS1 interacted with various miRNAs to modulate cancer development, such as miR‐186,^14^ miR‐99a/miR‐449a,^15^ miR‐125a,^16^ miR‐323,^17^ and so on.

In the present study, we showed that CDKN2B‐AS1 was overexpressed in cervical cancer and it might play an oncogenic role in promoting malignancy of cervical cancer cells, including proliferation promotion, apoptosis inhibition, and senescence inhibition. Importantly, our mechanistic analysis revealed that CDKN2B‐AS1 might function as an endogenous sponge to upregulate the expression of TGFβI through directly interacting and inhibiting the expression of miR‐181a‐5p. Our results provide a novel CDKN2B‐AS1/miR‐181a‐5p/TGFβI axis in the regulation of cervical cancer, shedding new light on the diagnosis and treatment for cervical cancer.

## 2 MATERIALS AND METHODS

### 2.1 Cell culture

The human cervical normal cell line Etc1/E6E7 and cancer cell lines (HeLa, C4‐1, SiHa, Ca Ski cells) were purchased from the American type culture collection (ATCC; Manassas, VA). Etc1/E6E7 cells were grown in Keratinocyte‐Serum Free medium (Gibco, Carlsbad, CA) with 0.1 ng/mL human recombinant EGF, 0.05 mg/mL bovine pituitary extract, and additional calcium chloride 44.1 mg/L (final concentration 0.4 mM). HeLa, C4‐1, SiHa, and Ca Ski cells were grown separately in Eagle's Minimum Essential Medium(EMEM, Gibco), Waymouth's MB 752/1 medium (Gibco), EMEM (Gibco), and RPMI‐1640 Medium (Gibco) complemented with 10% FBS (Life Technologies, Grand Island), and all cell lines were incubated at 37°C in a 5% CO2 incubator.

### 2.2 Quantitative real‐time polymerase chain reaction (qRT‐PCR)

Total RNA was extracted from cells using TRIzol reagent (Invitrogen, Carlsbad) according to the manufacturer's protocol. Equal amounts of RNA were reversely transcribed to cDNA with SuperScript Reverse Transcriptase Kit (Vazyme, Nanjing, China). Then mRNA levels of miR‐181a, TGFβI, and CDKN2B‐AS1 were analyzed by SYBR Green PCR Master Mix (Vazyme) in a Fast Real‐time PCR 7300 System (Applied Biosystems, Foster City). Data were analyzed according to the comparative Ct method also referred to as the 2^−ΔΔCT^ method. The expression level of miR‐181a‐5p was performed using miR‐181a‐5P‐specific primer. miR‐181a was normalized to snRNA U6, TGFβI and CDKN2B‐AS1 were normalized to GAPDH.

### 2.3 Cell transfection

CDKN2B‐AS1 small hairpin (Sh‐CDKN2B‐AS1)/negative control shRNA plasmids were purchased from Genechem, Shanghai, China. The miR‐181a‐5p inhibitor used in the experiment was designed and synthesized by Ribobio (Guangzhou, China). The HeLa cells were seeded in 6‐well plates at a density of 1×10^4^ cells/mL. After incubation for 24 hours, Sh‐CDKN2B‐AS1, adenovirus packaging vector‐CDKN2B‐AS1 (Ad‐CDKN2B‐AS1) and miR‐181a‐5p inhibitor were transfected into HeLa cell line by using Lipofectamine® 3000 (Invitrogen, USA) according to the instructions. The negative control shRNA was used as a control.

### 2.4 Western blot

Cells and tumor specimens were lysed with RIPA Lysis Buffer (Beyotime Institute of Biotechnology). Equivalent amounts of protein sample were separated by 10% SDS‐PAGE and transferred to PVDF membranes (Millipore, Billerica, MA). After incubated with 5% skim milk in TBST, the membranes were incubated with rabbit primary antibodies (Abcam, Cambridge, MA) against TGFβI (ab170874), VEGFA (ab52917), Vimentin (ab92547), Ki67 (ab16667), cleaved caspase‐3 (ab13847), E‐cadherin (ab40772), N‐cadherin (ab76011), and Snail (ab82846), respectively at 4℃ overnight. Then, incubated with HRP‐conjugated secondary antibodies (ab6721) at room temperature for 1.5 hours. Finally, the blots were visualized by ECL and detected using a ChemiDoc XRS imaging system. GAPDH was used as a loading control.

### 2.5 Luciferase reporter assay

The 3’UTR of CDKN2B‐AS1 mRNA containing predicted miR‐181a binding sites or mutant binding sites was PCR‐amplified and inserted into pMIR‐control vectors. For luciferase reporter assays, wild‐type or mutated versions of reporter plasmids, miR‐181a mimics were transfected into HEK 293 T by Lipofectamine 3000 regent. At 48 hours after transfection, the luciferase activities were measured with a dual luciferase reporter assay system (Promega, WI) according to the manufacturer's instructions. Data were normalized to Renilla activity.

### 2.6 Migration and transwell invasion assay

HeLa cells transfected with Sh‐CDKN2B‐AS1 or miR‐181a‐5p inhibitor or Ad‐CDKN2B‐AS1 were cultured in a 24‐well chamber. The confluent cell monolayer was scraped with a pipette tip in the middle of the well. After 24 hours of incubation, the cell migration was captured with a DM2500 bright field microscope (LEICA, Wetzlar, Germany) and the migration distance was measured by the ImageJ software.

The invasion capacity of HeLa cells was performed using Transwell invasion assay. Briefly, cells transfected with Sh‐CDKN2B‐AS1 or miR‐181a‐5p inhibitor or Ad‐CDKN2B‐AS1 were seeded in the upper chamber in EMEM supplemented with 0.1% FBS, and the lower chamber was filled with EMEM supplemented with 10% FBS. After 24 hours of incubation, the bottom cells were fixed in 95% ethanol, stained with hematoxylin, and the number of invaded cells was counted by using a DM2500 bright field microscope at 400 × magnification on 10 random fields in each well.

### 2.7 Hoechst 33258 assay for apoptosis

HeLa cells transfected with Sh‐CDKN2B‐AS1 or miR‐181a‐5p inhibitor were cultured in a 24‐well chamber. Then, the apoptosis of cells was detected by using Hoechst 33258 staining (Beyotime Institute of Biotechnology; C0003). The HeLa cells were fixed in 0.5 mL methanol for 30 minutes and washed with PBS three times. Next, the cells were dyed with 0.5 mL Hoechst 33258 for 10 minutes at room temperature in the dark place and washed for three times. The apoptotic cells were distinguished by cell morphological changes, such as chromatin condensation, nuclear fragmentation, and the cells were stained bright blue by hoechst. In each group, 10 random microscopic fields were examined and photographed under a fluorescence microscope (OLYMPUS, Japan). Subsequently, the apoptosis rate was quantified.

### 2.8 β‑galactosidase senescence assays

A total of 1 × 10^6^ HeLa cells were cultured in a 6‑cm dish and incubated for 3 days in EMEM medium supplemented with 10% FBS. When the cells reached approximately 80% confluence, they were fixed and incubated with a freshly prepared senescence‑associated β‑galactosidase staining solution in the dark at 37°C overnight. The percentage of cells that were positive for β‑galactosidase activity was determined by counting the number of blue cells in 10 fields at 20 × magnification. Each experiment was repeated three times.

### 2.9 Animal experimental protocols

Four‐week‐old female BALB/c nude mice were obtained from the Henan Laboratory Animal Center (Henan, China). A total of 20 animals were equally divided into two groups: One group was injected subcutaneously with 5×10^6^ HeLa cells which was transfected with Sh‐CDKN2B‐AS1, and another group was injected with scrambled HeLa cells. The HeLa cells were injected subcutaneously into the flanks of each 4‐week‐old BALB/c nude mice and fed for 30 days. Mice were housed under standard conditions (25 ± 2°C, 70% humidity and 12‐hour light‐dark periods) and fed on regular sterile chow diet and water ad libitum. All the animal experiments were performed in accordance with the National Institutes of Health guide for the care and use of Laboratory animals, and the protocols were pre‐approved by the Animal Care and Use Committee. The weight of all tumors was weighed after all mice were sacrificed.

### 2.10 Immunohistochemistry

The paraffin‐embedded tumor sections were stained for anti‐Ki67 and anti‐caspase‐3 (Abcam). Sections (2 μm) were deparaffinized and pretreated with citrate buffer using a heat‐induced epitope retrieval protocol. Endogenous peroxidase was blocked with 20% hydrogen peroxide for 15 minutes at room temperature followed by incubation with anti‐Ki67, and anti‐caspase‐3 for 30 minutes, respectively. A biotinylated goat anti‐mouse immunoglobulin G secondary antibody (Dako, Denmark) was then applied to each slide for 30 minutes. After washing in Tris‐hydrochloric acid buffer (TBS), the slides were incubated with peroxidase‐conjugated streptavidin complex reagent (Dako) and developed with 3,3’‐diaminobenzidine for 5 minutes. The slides were counterstained and dehydrated. Positive cells were detected as a brown staining. The treated specimens were observed and analyzed by using a microscope (OLYMPUS, Japan).

### 2.11 Bioinformatics data set

Prediction of the interaction between miR‐181a and TGFβI or CDKN2B‐AS1 was performed using miRnada (http://www.microrna.org) and TargetScan (http://www.targetscan.org).

### 2.12 Statistical analysis

The data were presented as mean ±standard deviation (SD) and analyzed using variance (ANOVA) test, student's t test, and linear regression test that were a part of the SPSS software (version 19.0). Values of *P* < 0.05 were considered statistically significant.

## 3 RESULTS

### 3.1 CDKN2B‐AS1 and miR‐181a‐5p is dysregulated in human cervical cancer

To investigate the role of CDKN2B‐AS1 and miR‐181a‐5p in cervical cancer progression, we determined the expression level of CDKN2B‐AS1 and miR‐181a‐5p in human normal cervical cell line Etc1/E6E7 and in cervical cancer lines HeLa, C4‐1, SiHa, and Ca Ski cells. As a result, we found that the expression level of CDKN2B‐AS1 was significantly higher than that in normal Etc1/E6E7 cells, including C4‐1 (*P < 0.01*), SiHa (*P < 0.05*), Ca Ski (*P < 0.05*), especially HeLa cells (*P < 0.001*) cells (Figure 1A), while the expression level of miR‐181a‐5p was significantly lower than that in normal Etc1/E6E7 cells, including C4‐1 (*P < 0.01*), SiHa (*P < 0.05*), Ca Ski (*P < 0.05*), especially HeLa cells (*P < 0.001*) cells (Figure 1B).

**Figure 1:** CDKN2B‐AS1 was upregulated and miR‐181a‐5p was downregulated in cervical cancer cell lines. (A) CDKN2B‐AS1 expression was detected in human cervical normal cell line Etc1/E6E7 and HPV‐18 infected cervical cancer cells HeLa, C4‐1 as well as HPV‐16‐infected cervical cancer cells SiHa, Ca Ski by qRT‐PCR. GAPDH was used as the internal control. *P < 0.05, **P < 0.01, ***P < 0.001, compared with Etc1/E6E7 group. (B) miR‐181a‐5p expression was detected in human normal cervical cell line Etc1/E6E7 and in cervical cancer lines HeLa, C4‐1, SiHa and Ca Ski cells by qRT‐PCR. U6 was used as the internal control. *P < 0.05, **P < 0.01, ***P < 0.001 compared with Etc1/E6E7 group

### 3.2 miR‐181a‐5p is a target of CDKN2B‐AS1

Since the inverse expression trend between CDKN2B‐AS1 and miR‐181a‐5p was observed in cervical cancer cells (Figure 1), we further studied whether there were direct interactions between them. Prediction of miR‐181a‐5p target sites was performed by the online software miRnada Tools. As shown in Figure 2A, CDKN2B‐AS1 contains many elements complementary to miR‐181a‐5p regions. The expression levels of miR‐181a‐5p were measured in Sh‐CDKN2B‐AS1 transfected HeLa cells by qRT‐PCR. miR‐181a‐5p inhibitor was introduced to identify the interaction between CDKN2B‐AS1 and miR‐181a‐5p. Expectedly, the expression levels of miR‐181a‐5p were markedly elevated in Sh‐CDKN2B‐AS1 group compared with the control group (*P < 0.01*), while miR‐181a‐5p inhibitor group showed decreased expression level of miR‐181a‐5p compared with the control group (*P < 0.01*), meanwhile, co‐transfection of Sh‐CDKN2B‐AS1 and miR‐181a‐5p inhibitor exhibited a middle expression level of miR‐181a‐5p (Figure 2B). Reversely, overexpression of CDKN2B‐AS1(Ad‐CDKN2B‐AS1) significantly reduced the expression of miR‐181a‐5p compared with the control group (*P < 0.01*), while miR‐181a‐5p mimic transfection decreased the expression level of miR‐181a‐5p compared with the control group (*P < 0.01*), meanwhile, co‐transfection of Sh‐CDKN2B‐AS1 and miR‐181a‐5p inhibitor exhibited a middle expression level of miR‐181a‐5p (Figure 2C). Bioinformatics and qRT‐PCR results revealed that CDKN2B‐AS1 interacted with miR‐181a‐5p and downregulates its expression in HeLa cells. To confirm this possibility, the wild type sequence of CDKN2B‐AS1 (CDK‐wt) or its mutant sequence (CDK‐mut) was subcloned into the pMIR luciferase reporter and then co‐transfected with miR‐181a‐5p mimics or controls into HeLa cells. As shown in Figure 2D, miR‐181a‐5p reduced luciferase activity in cells transfected with CDK‐wt (*P < 0.01*), but no effects were observed in cells transfected with CDKN2B‐AS1‐mut. These results indicated that there existed direct interactions between miR‐181a‐5p and the miRNA recognition sites of CDKN2B‐AS1.

**Figure 2:** CDKN2B‐AS1 can directly interact with miR‐181a‐5p in HeLa cells. (A) Predict binding sites between CDKN2B‐AS1 and miR‐181a‐5p. (B) The expression of miR‐181a‐5p mRNA level was detected in HeLa cells after sh‐CDKN2B‐AS1 transfection with or without miR‐181a inhibitor by qRT‐PCR. U6 was used as the internal control. **P < 0.01, compared with control group. ##*P < 0.01*, compared with miR‐181a inhibitor group. (C) CDKN2B‐AS1 was constructed on adenovirus packaging vector (Ad‐CDKN2B‐AS1). The expression of miR‐181a‐5p mRNA level was detected in HeLa cells after Ad‐CDKN2B‐AS1 transfection with or without miR‐181a mimic by qRT‐PCR. U6 was used as the internal control. **P < 0.01, compared with control group. ##*P < 0.01*, compared with miR‐181a mimic group. (D) Luciferase activity was detected by Luciferase reporter assay. HEK 293 T cells were co‐transfected with either 50 nM miR‐181a‐5p mimics or NC oligos and 200 ng of pmirGLO‐CDK‐wt or pmirGLO‐CDK‐mut using Lipofectamine 2000. The relative firefly luciferase activity was measured 24 hours after transfection and was normalized with renilla luciferase activity ^&&^ *P < 0.01* compared with CDK‐wt group. The data shown are the mean ± standard error of three individual experiments. CDK = CDKN2B‐AS1

### 3.3 CDKN2B‐AS1 knockdown suppresses migration and invasion of HeLa cells via derepression of miR‐181a‐5p

To further investigate the roles of CDKN2B‐AS1 and miR‐181a‐5p in HeLa cells,Sh‐CDKN2B‐AS1 and miR‐181a‐5p inhibitor were performed in transwell assay and wound healing assay. miR‐181a‐5p inhibitor was introduced to interfere the expression of miR‐181a‐5p. Transwell assay results showed that CDKN2B‐AS1 knockdown significantly inhibited the invasion of HeLa cells, while miR‐181a‐5p inhibitor obviously promoted the invasion of HeLa cells (Figure 3A, *P < 0.01*). What's more, wound healing results showed that CDKN2B‐AS1 knockdown significantly inhibited the migration of HeLa cells, while miR‐181a‐5p inhibitor obviously promoted the migration of HeLa cells (Figure 3B, *P < 0.01*). Besides, the combination of Sh‐CDKN2B‐AS1 and miR‐181a‐5p inhibitor exhibited a subdued activity compared with miR‐181a‐5p inhibitor alone, which suggested that CDKN2B‐AS1 knockdown suppressed migration and invasion of HeLa cells via derepression of miR‐181a‐5p.

**Figure 3:** CDKN2B‐AS1 contributed to invasion and migration of HeLa cells by inhibiting miR‐181a‐5p. Cells were divided into four groups: Ctrl, sh‐CDKN2B‐AS1, miR‐181a inhibitor, sh‐CDK +inhibi inhibitor. (A) The invasion abilities of HeLa cells were detected by Boyden Chamber Transwell assays. The cell invasion abilities were quantified. Mean cell counts from at least 10 fields and data represent the mean ± SD of triplicate determinations from three separate experiments and compared using the unpaired *t* test. (B) The migration abilities of HeLa cells were detected by wound healing assays. HeLa cells scraped by a pipette tip were cultured for 24 h. A representative of wound healing assay was presented. **P < 0.01, compared with Ctrl group. ^##^ *P* < 0.01, compared with miR‐181a inhibitor group

### 3.4 CDKN2B‐AS1 knockdown reduces EMT in HeLa cells via derepression of miR‐181a‐5p

The effects of CDKN2B‐AS1 knockdown on EMT were determined by measuring EMT mark proteins including E‐cadherin, N‐cadherin, Vimentin and Snail. As shown in Figure 4, compared to the control group, the protein expressions of E‐cadherin were significantly decreased in Sh‐CDKN2B‐AS1 group. It was demonstrated that Sh‐CDKN2B‐AS1 could enhance the expressions of N‐cadherin, Vimentin and Snail, while miR‐181a‐5p inhibitor showed opposite effects (Figure 4, *P < 0.01*). These results indicated that Sh‐CDKN2B‐AS1 could reduce EMT in HeLa cells via derepression of miR‐181a‐5p.

**Figure 4:** CDKN2B‐AS1 knockdown suppressed EMT of HeLa cells. The relative protein expression of E‐cadherin, Vimentin, N‐cadherin, and Snail were detected in HeLa cells after sh‐CDKN2B‐AS1 transfection with or without miR‐181a inhibitor by western blot. GAPDH was used as internal control. **P < 0.01, compared with control group. ##*P* < 0.01, compared with miR‐181a inhibitor group

### 3.5 CDKN2B‐AS1 knockdown inhibits proliferation and promotes apoptosis and senescence of HeLa cells via derepression of miR‐181a‐5p

The effects of CDKN2B‐AS1 knockdown on apoptosis was investigated by Hoechst staining. As shown in Figure 5A, the Sh‐CDKN2B‐AS1 transfection increased the apoptosis, while miR‐181a‐5p inhibitor transfection significantly decreased the apoptosis. Besides, the protein expression levels of Ki67 were downregulated by Sh‐CDKN2B‐AS1 transfection and cleaved caspase‐3 were upregulated by Sh‐CDKN2B‐AS1 transfection. Similarly, miR‐181a‐5p inhibitor showed opposite effects (Figure 5B, *P < 0.01*). Moreover, β‑galactosidase senescence assays showed that Sh‐CDKN2B‐AS1 transfection significantly increased the senescent cells and miR‐181a‐5p inhibitor obviously reduced the senescent cells(Figure 5C, *P < 0.01*). Interestingly, the combination of Sh‐CDKN2B‐AS1 and miR‐181a‐5p inhibitor exhibited a subdued activity compared with miR‐181a‐5p inhibitor alone, which suggested that Sh‐CDKN2B‐AS1 played roles (apoptosis induction, proliferation inhibition, and senescence induction) in HeLa cells via derepression of miR‐181a‐5p.

**Figure 5:** CDKN2B‐AS1 knockdown suppressed proliferation and promoted apoptosis and senescence of HeLa cells. Cells were divided into four groups: Ctrl, sh‐CDKN2B‐AS1, miR‐181a inhibitor, sh‐CDK +inhibi inhibitor. (A) Hoechst Staining and apoptosis rate were quantified. (C) Protein expressions of Ki67 and cleaved Caspase‐3, GAPDH acted as an internal control. Quantitation of signal intensities was performed by ImageJ software. (D) Senescence was detected by Senescence β‐Galactosidase Staining Kit

### 3.6 miR‐181a‐5p suppression regulated EMT, apoptosis and senescence via targeting TGFβI

Prediction of miR‐181a‐5p target sites was performed by the online software miRnada Tools. As shown in Figure 6A, TGFβI contains many elements complementary to miR‐181a‐5p regions. The expression levels of TGFβI were measured in human normal cervical cell line Etc1/E6E7 and in cervical cancer lines HeLa, C4‐1, SiHa, and Ca Ski cells. The mRNA level of TGFβI exhibited similar results with CDKN2B‐AS1 (Figure 6B). 10 μM SB431542 (selleckchem, Houston, USA; cat. no. S1067) and Ad‐CDKN2B‐AS1 were introduced to perform the experiments. According to the previous results, as shown in Figure 6C, Ad‐CDKN2B‐AS1 significantly increased the expression of TGFΒI, VEGFA, and Vimentin, while SB431542 played the opposite role (Figure 6C). Moreover, Ad‐CDKN2B‐AS1 increased the invasive cells (Figure 6D) but decreased the apoptosis rate (Figure 6E) and senescent cells (Figure 6F). Similarly, SB431542 exhibited reversed activity (Figure 6D‐F). These results confirmed that the TGFΒI was a target of miR‐181a‐5p and CDKN2B‐AS1 overexpression activated TGFΒI/VEGFA signal.

**Figure 6:** miR‐181a‐5p regulated EMT, apoptosis and senescence via targeting TGFβI. (A) Predict binding sites between TGFβI and miR‐181a‐5p. (B) TGFβI expression was detected in human normal cervical cell line Etc1/E6E7 and in cervical cancer lines HeLa, C4‐1, SiHa and Ca Ski cells by qRT‐PCR. GAPDH was used as the internal control. ^*^P < 0.05,^**^P < 0.01, ^***^P < 0.001 compared with Etc1/E6E7 group. (C) SB431542 was introduced to inhibit TGFβI. HeLa cells were transfected with Ad‐CDKN2B‐AS1 with or without SB431542. The relative protein levels of TGFβI, VEGFA, and Vimentin were detected in HeLa cells by western blot. GAPDH was used as internal control. (D) The cell invasion abilities were quantified. (E) Apoptosis rate was quantified. (F) Senescence was detected by Senescence β‐Galactosidase Staining Kit. **P < 0.01, compared with Ctrl group. ##*P < 0.01*, compared with SB431542 group.

### 3.7 *CDKN2B‐AS1 knockdown inhibits cell growth, EMT*,* and induced apoptosis* in vivo

Our previous in vitro studies have shown that CDKN2B‐AS1 knockdown suppressed growth and EMT, while CDKN2B‐AS1 knockdown promoted apoptosis in cervical cancer cells. We therefore studied the effects of CDKN2B‐AS1 in HeLa cell xenografted tumor mice in vivo. Consistent with the results in vitro, sh‐CDKN2B‐AS1 markedly suppressed the tumor weight compared to the control (*P < 0.01,* Figure 7A). Obviously, sh‐CDKN2B‐AS1 downregulated the mRNA level of CDKN2B‐AS1 but upregulated the mRNA level of miR‐181a‐5p (*P *< 0.01*,* Figure 7B). In addition, sh‐CDKN2B‐AS1 downregulated the protein levels of TGFβI, VEGFA, and Vimentin, which indicated that CDKN2B‐AS1 knockdown suppressed EMT in vivo(*P *< 0.01*,* Figure 7C). The immunohistochemistry results showed that CDKN2B‐AS1 knockdown decreased the expression of Ki67 and increased the expression of caspase‐3 in vivo (*P* < 0.01, Figure 7D). The results supplemented the anticancer activity of miR‐181a‐5p in vivo.

**Figure 7:** CDKN2B‐AS1 knockdown suppressed HeLa xenografted tumor survival in vivo. (A) sh‐CDKN2B‐AS1 decreased tumor weight. **P < 0.01 compared with control group. (B) The relative expression of CDKN2B‐AS1 and miR‐181a‐5p in HeLa(with or without sh‐CDKN2B‐AS1 transfection) xenografted tumor.(C) The relative protein levels of TGFβI, VEGFA, and Vimentin were detected in HeLa(with or without sh‐CDKN2B‐AS1 transfection) xenografted tumors by western blot. GAPDH was used as internal control. (D) The protein expression of caspase‐3 and Ki67 was detected by immunohistochemistry. Positive cells were counted. The data shown are the mean ± standard error of three individual experiments. ***P < 0.001, compared with control group

## 4 DISCUSSION

LncRNA CDKN2B‐AS1 has been studied well in many cancers. For example, CDKN2B‐AS1 was reported to promote proliferation and inhibit apoptosis in hepatocellular carcinoma,^9^ non‐small cell lung cancer,^10^ and bladder cancer.^12^ It is a common strategy to kill cancer by suppressing cancer cell proliferation and inducing apoptosis. The present study has supplemented the tumorigenic role of CDKN2B‐AS1 in cervical cancer. Meanwhile, CDKN2B‐AS1 knockdown resulted in proliferation inhibition and apoptosis induction. Invasion and migration are targets of cancer cells in cancer treatment. CDKN2B‐AS1 contributed to invasion and migration promotion in numerous cancers as reported in ovarian cancer,^11^ thyroid cancer,^18^ lung cancer, and 19 colorectal cancer.^20^ There are several researches that have discussed the tumorigenic role of CDKN2B‐AS1 in cervical cancer.^10^, ^14^, ^21^, ^22^ Moreover, CDKN2B‐AS1 was reported to inhibit senescence in epithelial ovarian cancer.^13^ Consistent with the previous results, our data showed that CDKN2B‐AS1 overexpression contributed to cervical cancer development by modulating the proliferation, apoptosis, invasion, migration, EMT and senescence, while CDKN2B‐AS1 knockdown showed totally reversed effects.

Increasing evidences demonstrated that miR‐181a‐5p have tumor‐suppressive functions. miR‐181a‐5p was observed with low expression in non‐small cell lung cancer,^23^ hepatocellular carcinoma,^24^ gastric cancer,^25^ ovarian cancer,^26^ and colorectal cancer.^27^ Most of the aforementioned studies demonstrated that miR‐181a‐5p inhibited cell proliferation and migration.^23^, ^27^ Others reported that lncRNAs may interact with miR‐181a‐5p to modulate cancer progression, such as CRNDE, MEG2, ZEB1‐AS1, and CCAT1.^25^, ^27^, ^28^, ^29^ Our study showed that miR‐181a‐5p was downregulated in cervical cancer cells. Importantly, miR‐181a‐5p was a target of CDKN2B‐AS1 and the regulatory role of CDKN2B‐AS1 in cervical cancer was executed by sponging miR‐181a‐5p.

To study the mechanism of miR‐181a‐5p inhibiting cervical cancer cell metastasis, we combined the gene sequencing data with prediction software. TGFβI, an extracellular matrix protein, has been proved to promote integrin‐dependent cell adhesion and motility.^30^ Accumulating evidences showed that TGFβI exhibited tumorigenic roles in several cancers, such as colorectal cancer,^31^ prostate cancer,^32^ and nasopharyngeal carcinoma.^33^ Interestingly, the depletion of TGFβI by miRNA may result in migration suppression^32^ and drug resistance reduction.^33^ The relationship between cancer metastasis and TGFβI is further supported by evidence that TGFβI enhanced the metastatic properties of colon cancer cells in vivo and TGFβI promoted migration and invasion of renal cell carcinoma.^34^, ^35^ In the present study, higher expression of TGFβI in cervical cancer cell lines might imply its oncogenic role in cervical cancer. Furthermore, miR‐181a‐5p directly bounds to 3’UTR of TGFβI mRNA and miR‐181a‐5p in HeLa cells decreased the expression of TGFβI at protein levels, suggesting that TGFβI is a potential target of miR‐181a‐5p.

The present study showed that interference of CDKN2B‐AS1 restrained the migration and invasion of HeLa cells, while the interference of CDKN2B‐AS1 promoted the apoptosis and senescence of HeLa cells. In conclusion, our in vitro and in vivo results revealed that lncRNA CDKN2B‐AS1 may involve in the progression of cervical cancer and this regulation may be played through the miR‐181a‐5p/TGFβI axis. Our experimental data also suggested that the CDKN2B‐AS1/miR‐181a‐5p/TGFβI axis may be a promising therapeutic target for cervical cancer or other cancers.

## CONFLICTS OF INTEREST

The authors declare no competing interests.
